# Hippocampus Segmentation Method Based on Subspace Patch-Sparsity Clustering in Noisy Brain MRI

**DOI:** 10.1155/2021/3937222

**Published:** 2021-09-25

**Authors:** Xiaogang Ren, Yue Wu, Zhiying Cao

**Affiliations:** ^1^Changshu Hospital of Chinese Medicine, Changshu 215516, Jiangsu, China; ^2^School of Information and Control Engineering, China University of Mining and Technology, Xuzhou, Jiangsu 221116, China; ^3^The Affiliated Changshu Hospital of Soochow University (Changshu No. 1 People's Hospital), Suzhou, Jiangsu 215500, China

## Abstract

Since the hippocampus is of small size, low contrast, and irregular shape, a novel hippocampus segmentation method based on subspace patch-sparsity clustering in brain MRI is proposed to improve the segmentation accuracy, which requires that the representation coefficients in different subspaces should be as sparse as possible, while the representation coefficients in the same subspace should be as average as possible. By restraining the coefficient matrix with the patch-sparse constraint, the coefficient matrix contains a patch-sparse structure, which is helpful to the hippocampus segmentation. The experimental results show that our proposed method is effective in the noisy brain MRI data, which can well deal with hippocampus segmentation problem.

## 1. Introduction

The hippocampus is a decisive organization in the structure of human brain. Its function is to control memory and emotion and determine the spatial position [1]. As we all know, short-term memory is stored in the hippocampus. If the hippocampus is damaged, it will directly lead to partial or total irreversible loss of memory function [2]. The abnormal function and morphology of hippocampus may induce Alzheimer's disease [3], schizophrenia, temporal lobe epilepsy, severe depression, and other nervous system diseases [4]. Therefore, if the hippocampus can be accurately segmented from the brain tissue, it will be better to provide more accurate diagnostic basis for disease research, as shown in Figure 1 [5].

The difficulty of image segmentation is that there are many kinds of images with different quality, so it is impossible to establish a unified image segmentation standard [6]. How to segment the image quickly and effectively has always been the focus of image processing. So far, there is no general method of accurate image segmentation, but the cognition of image segmentation has become more and more clear, and many image segmentation methods have been produced. Different segmentation methods generally understand the problem of image segmentation from different perspectives.

The hippocampus has the characteristics of small size and irregular shape. The traditional segmentation method is prone to the wrong segmentation, and the segmentation speed is slow, which consumes a lot of time. In order to solve various problems in the process of hippocampus segmentation, the development of segmentation technology is mainly divided into manual segmentation, semiautomatic segmentation, and automatic segmentation [5]. Manual segmentation refers to experienced clinicians directly drawing the boundary of the hippocampus on the brain MRI image or drawing the boundary of the relevant tissues on the computer display through the mouse to form the region of interest. At present, the main purpose of hippocampus segmentation is to separate the interested objects from the brain MRI image background, so as to further analyze and recognize them quantitatively and understand the brain MRI image [5]. Due to the extremely complex diversity of medical images and the noise introduced in the brain MRI imaging equipment, there is a certain degree of noise in medical images, and some edges of the hippocampus object may not be clear [7]. Therefore, there is no general theory and method in hippocampus segmentation of brain MRI. The result of manual segmentation is usually regarded as the gold standard because of its high accuracy, but it is time-consuming and laborious at the same time [8]. The quality of the segmentation result completely depends on the operator's experience and knowledge, and the segmentation result is difficult to reproduce. Automatic segmentation means that the whole process of image segmentation is completely controlled by the computer and completely separated from the manual interference. Although this method can reproduce the segmentation results well, the computational complexity is also very large, and it requires high configuration of computer equipment. With the development of computer science and technology, the semiautomatic segmentation of human–computer combination model, also known as interactive segmentation method, comes into being [9]. It combines the experience of human knowledge with the powerful data processing, storage, and memory ability of computer and realizes image segmentation through human–computer interaction. However, the results of computer automatic segmentation are often not satisfactory, and the accuracy cannot meet the requirements of clinical application of medical images, while the manual segmentation, which relies too much on human experience, is also unacceptable in practical application [10]. The commonly used methods of hippocampal segmentation are threshold method, edge detection, region growing method, fuzzy clustering method [11, 12], graph theory-based max-flow/min-cut method, deformation model, neural network method, genetic algorithm, and wavelet transform method [13], where region growing segmentation based on seed points and deformation model methods are all interactive segmentation methods. Because of the complexity of human body structure, fuzzy edge, and uneven gray level, the medical image is more difficult to segment than nature image. Therefore, it is particularly important to study the hippocampus segmentation methods of medical images in depth.

At present, domestic and foreign scholars have made further research and exploration on the automatic hippocampus segmentation. Lu and Luo [14] proposed a segmentation method based on multi-atlas, which used similar weighted voting and label bias correction to achieve almost automatic segmentation of hippocampus. Wu et al. [15] used statistical model for automatic segmentation of hippocampus in brain MRI images, which is suitable for routine analysis of large-scale hippocampal formation. Some scholars have integrated the automatic segmentation technology of brain tissue and developed corresponding software, such as FSL and FreeSurfer [16]. The FSL is a tool library developed by the Oxford University for analyzing brain MRI. The tool library includes first toolkit, which can realize the automatic segmentation of brain structure and the segmentation of hippocampus, brain stem, nucleus accumbens, and other tissues. The FreeSurfer is developed by the world-famous Harvard Medical School and MIT, which can solve the problem of brain 3D MRI image data and automatically segment the cortex and subcutaneous nuclei by using the gold-standard prior probability information estimation.

Because of the weak edge of the object region in hippocampus MRI image, the existing active contour sequence segmentation models often show an edge-false problem. So, a contour transfer evolution based a segmentation method is proposed [17], which combines the region-based model and edge model based perfectly and transfers the growth edge of the object region in the current image to the adjacent image as its initial contour. As a result, the new model reduces iteration times and improves the accuracy of the segmentation results, but the performance of segmentation for a hippocampus with a small size and irregular shape is poor. The hippocampus segmentation method based on graph theory can make good use of multiscale redundancy features and has good segmentation effect. However, there is no unified method and standard for how to describe the image as a graph and how to extract it more accurately, and the representation of graph will affect the result of hippocampus segmentation [18].

In this paper, a novel image segmentation method based on subspace clustering is proposed, which regards the superpixel as the point of the image and chooses the matrix of the superpixel as the projection dictionary. By restraining the coefficient matrix with the block-sparse constraint, the coefficient matrix contains a patch-sparse structure, which is helpful to the hippocampus segmentation. The experimental results show that our proposed method is effective to the noisy brain MRI data, which can well deal with the hippocampus segmentation problem.

## 2. Related Works

### 2.1. Subspace Clustering

Subspace clustering, also known as subspace segmentation, assumes that the data are distributed in the union set of several low-dimensional subspaces, which is the process of classifying the data into their subspaces in some way [19]. Through subspace clustering, the data from the same subspace can be classified into one class, and the relevant properties of the corresponding subspace can be extracted from the same kind of data. Subspace clustering is to classify the data belonging to the subspace *S*_*i*_ in the data matrix *X* to obtain a low-dimensional representation of the data and thereby obtain the dimension and base matrix of the subspace *S*_*i*_. When the number of subspaces is one, the subspace clustering problem is equivalent to the principal component analysis. Through principal component analysis, the principal information of the data matrix can be obtained, so as to obtain the low-dimensional representation of these data. The most common method to solve the principal component analysis is singular value decomposition (SVD). When the number of subspaces is greater than one, the dimension and basis matrix of subspace are unknown, and the interaction between different subspaces makes the information obtained from the observation data inaccurate, which increases the difficulty of subspace clustering. Therefore, many scholars often assume that different subspaces are independent or noninteractive when building the subspace clustering models.

The process of subspace clustering is shown in Figure 2. There are many methods to realize subspace clustering, including algebraic method, iterative method, statistical method, and spectral clustering method [20]. The theoretical basis of each method is different, and there are also great differences in the solution process. However, the clustering results are obtained/solved by solving the representation coefficient of data matrix *X* under a specific base matrix. The representative method is to use the matrix decomposition method and spectral clustering method. In order to get the feature representation of data matrix *X* in subspace, *X* can be written as *X*=*DA*, where *D* represents the dictionary, the basis matrix can be obtained by training dictionary or using the iterative updating process, and *A* represents the representation coefficient matrix of data matrix *X* under dictionary *D*. By adding appropriate constraints to the coefficient matrix or dictionary, the data can be more accurately projected into its subspace. In this paper, we mainly studied the subspace clustering method based on spectral clustering for brain MRI hippocampus image, where the graph theory is taken as the theoretical basis and the data as the vertices in the graph. Therefore, the similarity between the vertices can be obtained by solving *X*=*DA*. Thus, the adjacency matrix of the graph is obtained, the Laplacian matrix of the graph is constructed, and the clustering result is obtained from the Laplacian matrix of the graph using the spectral clustering method, thereby obtaining the clustering result of the data.

The purpose of subspace clustering is to classify data from different subspaces into their corresponding subspaces [14]. The key point is to get the correct representation of the data in the subspace. The subspace clustering method is based on graph theory, using spectral clustering method to cluster data. The biggest difference among subspace clustering and traditional graph theory-based clustering and spectral clustering is that subspace clustering starts from the source of the data, focuses on the representation of the data in the subspace, and obtains more accurate data, while the subspace representation of data can also be used for data analysis and other processing. In the subspace clustering process, the data is regarded as the vertices in the graph, the weight matrix or adjacency matrix of the graph is obtained by solving the representation coefficient of the data in the subspace, and the final clustering result is obtained by using the spectral clustering method. The realization of a process is based on the mathematical theory of graph theory. The clustering process of data is transformed into the cutting process of the vertices of the graph. The connectivity of the graph is used to show the relationship between different classes.

### 2.2. Sparse Representation

Sparse representation is a research hotspot in the field of image processing recently. Its purpose is to better reveal the essential characteristics by using the sparse property of signal or image in a specific space [21]. The sparse representation of signal can be achieved by constructing appropriate dictionary and sparsity requirement of coefficients. In other words, the signal can be represented by as few atoms as possible in the dictionary. The obtained nonzero coefficients can represent the main structure and characteristics of the signal. In order to reveal the more essential characteristics and get a more sparse representation of the signal, many scholars have done a lot of work in the construction of dictionaries. Through dictionary construction, the signal has the basis of sparse representation, and the common method is to constrain the coefficients by l0 or l1 norm so as to get sparse coefficients. Sparse representation has achieved good results in many applications, such as compressed sensing, denoising, superresolution reconstruction, and texture decomposition [22]. Sparse subspace clustering method combines sparse representation theory and subspace representation coefficients. The final result of subspace clustering is to classify the data in the same subspace. When the subspaces are independent of each other, the data belonging to a certain subspace is only composed of the baseline in this subspace. In other words, the representation coefficient of these data in other subspaces is zero. Therefore, as for high-dimensional data, the representation coefficients of data in low-dimensional subspace are sparse. The data in the same subspace only have representation coefficients in this subspace, which shows the same sparsity. By solving the sparsity constraint of representation coefficients, the sparsity of data representation coefficients is highlighted, which provides support for the correct clustering.

According to the structural characteristics of the analyzed signal, any given observed signal *y* ∈ *R*^*N*^ can be expressed in a parameterized way, which can construct the feature dictionary *D* ∈ *R*^*N*×*M*^. *d* ∈ *D* is the atom in dictionary and ‖*d*‖=1. Therefore, the projection of *y* on the atoms in the dictionary can be written as *c*=〈*y*, *d*〉. The standard formula of sparse representation problem can be denoted as follows:

(1) $$\begin{array}{c} x^{*}=\underset{x}{\arg\min}{\left\|y-dx\right\|}_{2}^{2}+\lambda {\left\|x\right\|}_{0}, \end{array}$$

where ‖*x*‖_0_ represents the number of nonzero elements in *x*; *λ* > 0 data, and each column *x*_*i*_ is an n-dimensional feature vector. These data come from the union of *K* independent subspaces {*S*_*c*_}_*c*=1_^*K*^ with unknown dimension {*r*_*c*_}_*c*=1_^*K*^. The purpose of subspace clustering is to reveal the subspace attributes of each data by clustering, and different classes correspond to different subspaces. If any data in the subspace can be represented as a linear combination of other data, the matrix *Z* can be used to construct the similarity matrix. In order to obtain the matrix *Z*, the following optimization problem can be solved:

(2) $$\begin{array}{c} \left\{\begin{array}{cc} \min & \Omega {\left(Z\right)}_{Z,E}+\lambda \Phi \left(E\right),\\ s.t. & X=XZ+E, \end{array}\right. \end{array}$$

where Ω(*Z*) and *C* are the constraints on *Z*; *E* is the error value or abnormal value; Φ(*E*) is the constraint function of *E*. In general, ‖*E*‖_*F*_^2^ is used for Gaussian noise, and ‖*E*‖_1_ is used for abnormal value. *λ* is a trade-off parameter. The main difference between different clustering methods is the selection of Ω(*Z*). A suitable Ω(*Z*) is designed so that the matrix *Z* obtained from the model satisfies the properties of sparsity between classes and consistency within classes.

## 3. Subspace Patch Sparsity for Clustering Segmentation

### 3.1. Motivation

In Section 2, it is assumed that the data matrix can be denoted as *X*=[*X*_1_, *X*_2_,…, *X*_*n*_] ∈ *R*^*M*×*N*^, where *X*_*i*_ ∈ *R*^*M*×*n*_*i*_^, (*i*=1,2,…, *n*) , comes from *n* independent linear subspaces *S*_*i*_. The subspace representation problem *X*=*XA* has a solution with patch diagonal structure. For the previously mentioned subspace clustering problem, when the data is only represented by some atoms from the same subspace, the information of the data belonging to the same subspace can be easily obtained through the representation coefficient. When the data matrix is arranged via the matrix *A*, the representation is shown as the patch diagonal structure of the coefficient matrix. Theoretically, the coefficient matrix *A* has a patch diagonal structure, which means that the adjacency matrix *W* in the graph constructed by *A* also has a block diagonal structure. The patch diagonalization of the adjacency matrix indicates that the vertices in the same block constitute a connected subgraph and are not connected with other connected subgraphs, while the vertices in the connected subgraph are data in the same subspace. Therefore, the block diagonal structure of coefficient matrix plays an important role in subspace clustering.

In order to obtain the coefficient matrix with block diagonal structure, sparse subspace clustering and low-rank subspace clustering introduce sparse and low-rank constraints into subspace representation, respectively. The sparse clustering model measures the sparsity of the coefficients by *l*_1_. The adaptive sparse representation makes the coefficient sparse matrix under the sparsity constraint block, which reflects the block diagonal structure. The low-rank subspace clustering model uses the kernel norm to constrain the rank of the coefficient matrix. The operation of the whole matrix makes the low-rank constraint better retain the global structure of the coefficient matrix than the sparse constraint. In addition, it is proved theoretically that the solution of the low-rank optimization problem has the block diagonal structure. Therefore, sparse and low rank can get the coefficient matrix with block diagonal structure. However, the coefficient matrix in sparse model has the block-sparse property, but the actual solution process is to calculate each column of coefficient separately, so the isolated calculation does not use the global patch-sparse structure of coefficient matrix.

Both sparse model and low-rank model constrain data in the same subspace. The sparse model takes advantage of the sparsity of data representation, while the low-rank model starts from the global structure of the matrix and makes full use of the correlation of the same subspace data. Combined with the idea of the sparse and low-rank model, the subspace representation of data should show sparsity between different subspaces. In other words, the patch representation of subspace is sparse, and the representation of different data should be closer in the same subspace, making full use of the correlation between data. Inspired by the previously mentioned analysis, this paper introduces the *l*_1,2_ norm constraint to establish the patch-sparse subspace clustering model, which considers the global relationship of data in the subspace while calculating the sparsity of the coefficients.

### 3.2. Patch-Sparsity Model

Let *R*={*K*_1_, *K*_2_,…, *K*_*n*_} be a division of {1,2,…, *n*}, where *K*_*i*_ corresponds to the subscript of data in subspace*S*_*i*_. For a column vector *x* in data matrix *X*, the following model is constructed:

(3) $$\begin{array}{c} \left\{\begin{array}{cc} \min & \sum_{K\in R}{\left\|\alpha_{k}\right\|}_{2},\\ s.t. & x=Xa, \end{array}\right. \end{array}$$

where *a*_*k*_ is a vector composed of elements whose subscripts belong to *k* in feature matrix *a* norm. Therefore, the solution of (3) can be equivalent to the solution of the following equation:

(4) $$\begin{array}{c} \underset{\alpha }{\min}{\left\|Xa-x\right\|}_{2}+\lambda \sum_{K\in R}{\left\|\alpha_{K}\right\|}_{2}, \end{array}$$

where *λ* is the regularization parameter and is typically set to 0.1.

For the sake of analysis, we can rewrite (4) as a matrix form, which can be denoted as follows:

(5) $$\begin{array}{c} \underset{\text{A}}{\text{min}}\frac{1}{2}{\left\|XA-X\right\|}_{F}^{2}+\lambda \sum_{j=1}^{N}\sum_{k\in R}{\left\|{\left(A_{j}\right)}_{k}\right\|}_{2}, \end{array}$$

where *A*=[*A*_1_, *A*_2_,…, *A*_*N*_] ∈ *R*^*N*×*N*^, and (*A*_*j*_)_*k*_ is the vector of elements that are subscript to *k*.

In order to obtain the solution of the model, we deduce it according to the following steps. As for *l*_1_ optimization problem $\underset{\alpha }{\min}{\left\|D\alpha -x\right\|}_{2}^{2}+\lambda {\left\|\alpha \right\|}_{1}$, least absolute shrinkage and selection operator (LASSO) can be adopted to obtain the optimal result. As for *l*_2_ optimization problem $\underset{\alpha }{\min}{\left\|D\alpha -x\right\|}_{2}^{2}+\lambda \sum_{k\in R}w_{k}{\left\|\alpha_{k}\right\|}_{2}$, group LASSO can be adopted, where *w*_*k*_ is the number of elements in each group. As for *l*_1,2_ optimization problem, some scholars introduced the block coordinate descent into group LASSO.

If the data patches, whose subscript set is *K*, are selected and other patches are fixed, (3) can be rewritten as follows:

(6) $$\begin{array}{c} \underset{\alpha_{\text{k}}}{\text{min}}\frac{1}{2}{\left\|X_{K}\alpha_{K}-x\right\|}_{2}^{2}+\lambda {\left\|\alpha_{K}\right\|}_{2}^{2}, \end{array}$$

where *k*_*i*_ is a matrix composed of column vectors whose subscripts belong to *K* in *X*. Through the patches threshold method, we can get the following:

(7) $$\begin{array}{c} \alpha_{k}=\left\{\begin{array}{cc} 0, & if\;{\left\|X_{K}^{T}x\right\|}_{2}\leq \lambda ,\\ {\left(X_{K}^{T}X_{K}+\delta \lambda I\right)}^{-1}X_{K}^{T}x, & if\;{\left\|X_{K}^{T}x\right\|}_{2}>\lambda , \end{array}\right. \end{array}$$

where *δ* > 0 and *δ*^−1^=‖(*X*_*K*_^*T*^*X*_*K*_+*δλI*)^−1^*X*_*K*_^*T*^*x*‖_2_ when ‖*X*_*K*_^*T*^*x*‖_2_ > *λ* is given.

If *δ* can satisfy *δ*^−1^=‖(*X*_*K*_^*T*^*X*_*K*_+*δλI*)^−1^*X*_*K*_^*T*^*x*‖_2_, *δ* is the root of the equation *f*(*δ*)=1. If $X_{K}^{T}X_{K}=\left[\begin{array}{ccc} \sigma_{1} & \cdots & 0\\ \vdots & \ddots & \vdots \\ 0 & \cdots & \sigma_{L} \end{array}\right]$ makes sense, we have

(8) $$\begin{array}{c} f\left(\delta \right)=\delta {\left\|{\left(X_{K}^{T}X_{K}+\delta \lambda I\right)}^{-1}X_{K}^{T}x\right\|}_{2}=\sqrt{\sum_{i}\frac{\delta^{2}{\left(X_{K}^{T}x\right)}_{i}^{2}}{{\left(\delta \lambda +\sigma_{i}\right)}^{2}},} \end{array}$$

where is the number of elements in *K*. When *δ*=0, we can get *f*(*δ*)=0; if *δ*⟶*∞* and ‖*X*_*K*_^*T*^*x*‖_2_ > *λ*, the following results can be obtained:

(9) $$\begin{array}{c} \underset{\delta ⟶\infty }{\lim}f\left(\delta \right)=\underset{\delta ⟶\infty }{\lim}\sqrt{\sum_{i}\frac{{\left(X_{K}^{T}x\right)}_{i}^{2}}{{\left(\lambda +\sigma_{i}/\delta \right)}^{2}}}=\sqrt{\sum_{i}\frac{{\left(X_{K}^{T}x\right)}_{i}^{2}}{\lambda }}>1. \end{array}$$

Thus, it is shown that there are solutions to *f*(*δ*)=1. It is assumed that the partition *K* is known, but in reality, the division *ℜ* is required to solve the subspace clustering problem. The closer the selection of division is to the real subspace division of the data, the closer the actual subspace representation is to the solution of equation (5). When *ℜ*, equation (4) becomes an *l*_1_ optimization problem, while equation (5) is transformed into a sparse model. It is worth noting that the division in *ℜ* often needs to be finer than the real division, which is to ensure that it is closer to the real division. Using some traditional clustering methods, such as *k*-means clustering, a preliminary division of the data can be obtained. In this paper, sparse agglomerative clustering (SAC) is adopted to determine the preliminary data division. In the construction of the block-sparse dictionary, the SAC algorithm can obtain the patch structure of the dictionary, which is the division of the dictionary atoms. The SAC algorithm introduces the index of the class and gradually merges the closest atoms to achieve the purpose of clustering. The clustering process does not need to define the number of classes but defines the upper bound of the number of elements in the class to limit the final clustering result.

## 4. Experimental Results and Analysis

### 4.1. Experimental Data and Configuration

In order to better show the advantages of the improved sparse subspace clustering segmentation method, this paper selects simulated brain MRI and real brain MRI data for simulation analysis. The real brain MRI data is 30 slices of 3D T1WI MRI images of adult male head with 3 mm slice provided by the Department of Radiology, West China Medical University. The simulation brain MRI is from the database BrainWeb, where BrainWeb provides standard segmentation results and is convenient for quantitative evaluation. It can help the validation of quantitative analyses of hippocampus.

The simulation platform uses MATLAB v7.8 (r2009a) and runs on core i5 processor with 8G memory and 2.94Ghz main frequency. The comparison algorithms used in this paper are sparse subspace clustering (SSC) [23], low-rank representation (LRR) [24], fuzzy GMM [25], LSM [26], and U-Net [27]. The first three models are the best algorithms in the traditional model, while U-Net is a semantic segmentation algorithm based on full convolution network, which is widely used in the field of natural image segmentation. In this paper, the contrast of brain MRI images is very low. The existing deep network algorithm is not adaptable. All comparison algorithms use the source code or executable file given by the author. It is worth noting that the test data selected in the experiment are the most challenging sequences available. In all experiments, all parameters of each algorithm are fixed to verify the robustness and stability of the proposed segmentation method. Therefore, in all experiments, if there is no special explanation, the parameters are set as follows: *c*_0_=2,  *u*=1, *λ*=10, *v*=0.05, *τ*=2,  and *σ*=1.

In order to qualitatively evaluate the performance of all the comparison algorithms, we use false negative ratio (FNR), ratio of segmentation error (RSE), and dice similarity coefficient (DSC) to measure the segmentation accuracy. It is assumed that *S*_1_ is denoted as the segmentation region obtained by each model and *S*_2_ is the real boundary of a given image, so the previously mentioned three evaluation criteria are defined as follows:

(10) $$\begin{array}{c} \text{FNR}=\frac{N\left(S_{1}/S_{2}\right)}{N\left(S_{1}\right)},\\ \text{RSE}=\frac{N\left(S_{1}/S_{2}\right)+N\left(S_{2}/S_{1}\right)}{N\left(\Omega \right)},\\ \text{DSC}=\frac{2N\left(S_{1}\cap S_{2}\right)}{N\left(S_{1}\right)+N\left(S_{2}\right)}, \end{array}$$

where *N*(*∗*) represents the number of pixels in the closed area. The closer the values of FNR and RSE are to zero and the closer the values of DSC are to one, the higher the image segmentation accuracy is.

### 4.2. Qualitative and Quantitative Analyses for Simulated Brain MRI

In order to better verify the effectiveness of the proposed method, it is tested on simulated brain MRI images and compared with the segmentation results of several classical algorithms. The data used in the experiment is from BrainWeb database. The test images were *T*1 weighted, 181 × 217 in size, and 1 mm in thickness. Before the experiment, extracranial tissues, such as blood vessels, cranium, and neuroticism, were removed and set as the background. In this paper, different slice images with added noise are selected as experimental data.  Figure 3 shows the segmentation result processed by different algorithms.

Figure 3(a) shows the original brain MR image; the image in Figure 3(b) adds Gaussian noise with a variance of 10; Figure 3(c) shows the standard segmentation results; Figures 3(c)–3(h) show the corresponding segmentation results of the comparison algorithm. Through the qualitative comparison of segmentation results, SSC and LRR methods cannot get satisfactory segmentation results, and there are obvious false segmentation points in fuzzy GMM and LSM. In contrast, the proposed model gets the best segmentation results among the five methods, especially in the boundary region and detail texture region. It can be seen from the segmentation result that, with the increase of noise, the segmentation accuracy of each algorithm decreases gradually. This is because the noise has a certain impact on the segmentation accuracy of brain image. The greater the noise is, the greater the texture change of brain image is, and the regions with more detail information are prone to partial misclassification. By comparing the five segmentation algorithms, we can see that the proposed algorithm can get the highest segmentation accuracy in the brain MR images of hippocampus under different noise levels.

It can be seen from the result that our proposed model uses the improved coefficient matrix with the patch-sparse constraint on brain MRI image. It can not only successfully extract the hippocampus tissue but also remove many misclassification points. The segmentation effect is obviously better than the other five comparison algorithms. By comparing with the standard segmentation results, the segmentation accuracy of each algorithm under different noises is given in Table 1. The experimental data are obtained by averaging for each slice under the same noise. It can be seen from the table that fuzzy-GMM algorithm achieves better segmentation effect under some conditions, and the segmentation accuracy of the proposed model is the highest in most cases. With the increase of noise level, the difference of FNR and RSE value of our model is very small, while the decrease of other comparison algorithms is obvious. The experimental results show that the noise has a great influence on the segmentation accuracy of brain MR images, and the larger the noise are, the easier it is to produce wrong classification. However, according to the results in Table 1, the proposed model is less affected by noise.

The previously mentioned analysis shows that the segmentation accuracy is different under different noises. In order to facilitate intuitive analysis, we draw three curves to show the segmentation results of different algorithms in Figure 4. The FNR, RSE, and DSC indexes of our proposed algorithm are better than those of other algorithms, especially DSC. In the general segmentation algorithm, when the contrast of the image becomes worse or the noise becomes larger, it is more difficult to distinguish the boundary of LSM from the anatomical characteristics of brain tissue. Therefore, the combination of sparsity and low rank is more effective than the general single model, which can reduce the impact of noise on segmentation and retain the corresponding details.

### 4.3. Qualitative and Quantitative Analyses for Real Brain MRI

The real brain MRI data is 30 slices of 3D T1WI MRI images of adult male head with 3 mm slice provided by the Department of Radiology, West China Medical University.  Table 2 shows the quantitative indicators of different algorithms. It can be seen that the segmentation performance for noisy images is not good. Although sparse and low-rank model is an effective processing strategy, it still has a shortcoming. First of all, the model requires sparse constraints on all image patches, which greatly reduces the real-time performance and improves the complexity of the model. The segmentation model proposed in this paper. LSM is an improved level-set model. From the analysis of segmentation effect, the traditional level-set method has the phenomenon of undersegmentation. This method only uses the gradient information of the image boundary, so the zero level-set curve is easy to stay in the nonobject region with large gradient value in the iterative process, which makes the final evolution result deviate from the real boundary of the hippocampus, and the hippocampus contour cannot be accurately segmented.

In order to quantitatively compare the segmentation performance on real brain MRI tissue, the real brain MRI database is used for experiments, which can provide the standard segmentation results, which is convenient to quantitatively evaluate the performance. *T*1 weighted brain MRI images with 1 mm slice thickness and 9% noise level are used as experimental data. In this paper, 20 slices in different positions are tested, and the segmentation result is shown. Due to the influence of space, we only give the segmentation results of our proposed algorithm, as shown in Figure 5. The segmentation results of fuzzy-GMM algorithm still contain a lot of noise. SSC algorithm, LRR algorithm, and proposed algorithm in this paper all remove the interference of noise very well. In terms of details, the proposed algorithm is the most complete for the preservation of the hippopotamus in brain MRI image.

Figure 6 shows the segmentation results of the comparison algorithm on the real brain MRI images.  Figure 6(a) is the original image; Figure 6(b) is the manually segmented hippocampus image; Figure 6(c) is the segmentation result obtained by the improved U-Net algorithm; Figure 6(d) is the segmentation result obtained by the fuzzy-GMM algorithm. The segmentation effect of our proposed subspace clustering segmentation is improved, and the segmentation result is the closest to that of manual annotation. The segmentation effect is the best, compared with other comparison algorithms in this paper. The sparse subspace clustering model SSC, low-rank subspace clustering model LRR, and block-sparse subspace in this paper are used.

## 5. Conclusion

Since the hippocampus is of small size, low contrast, and irregular shape, a novel hippocampus segmentation method based on subspace patch-sparsity clustering in brain MRI is proposed to improve the segmentation accuracy, which regards the super pixel as the point of the image and chooses the matrix of the super pixel as the projection dictionary. By restraining the coefficient matrix with the patch-sparse constraint, the coefficient matrix contains a patch-sparse structure, which is helpful to the hippocampus segmentation. The experimental results show that our proposed method is effective in the noisy brain MRI data, which can well deal with hippocampus segmentation problem.

## Figures and Tables

**Figure 1:** Example for hippocampus segmentation.

**Figure 2:** The process of subspace clustering.

**Figure 3:** Segmentation result of different algorithms: (a) raw MRI, (b) noisy MRI, (c) benchmark result, (d) fuzzy-GMM, (e) LSM, (f) SSC, (g) LRR, (h) U-Net, and (i) proposed.

**Figure 4:** Segmentation curves for (a) FNR, (b) RSE, and (c) DSC indexes in different noises.

**Figure 5:** Segmentation results of our proposed algorithm. (a) Raw data; (b) segmentation results.

**Figure 6:** Segmentation results of different algorithms. (a) Raw data, (b) benchmark result, (c) U-Net, (d) fuzzy-GMM, (e) SSC, (f) LRR, and (g) proposed.

**Table 1:** Quantitative results for comparison models in different noises.

*σ*		SSC	LRR	Fuzzy GMM	LSM	U-Net	Proposed
5	FNR	0.461	0.407	0.461	0.512	0.523	0.453
	RSE	0.082	0.089	0.099	0.182	0.181	0.089
	DSC	0.761	0.808	0.891	0.782	0.831	0.903

10	FNR	0.357	0.543	0.504	0.516	0.621	0.707
	RSE	0.075	0.087	0.098	0.078	0.086	0.060
	DSC	0.682	0.836	0.718	0.805	0.816	0.836

20	FNR	0.316	0.593	0.623	0.485	0.707	0.718
	RSE	0.068	0.067	0.070	0.072	0.074	0.064
	DSC	0.579	0.531	0.690	0.734	0.752	0.792

30	FNR	0.297	0.282	0.317	0.378	0.322	0.252
	RSE	0.050	0.063	0.052	0.036	0.060	0.044
	DSC	0.508	0.471	0.523	0.658	0.680	0.697

**Table 2:** Quantitative results for comparison models in real brain MRI.

	SSC	LRR	Fuzzy GMM	LSM	U-Net	Proposed
FNR	0.477	0.608	0.63	0.633	0.724	0.71
RSE	0.097	0.102	0.103	0.127	0.133	0.085
DSC	0.516	0.469	0.558	0.634	0.651	0.647

## Data Availability

The labeled datasets used to support the findings of this study are available from the corresponding author upon request.
